The article "High-rate aluminium yolk-shell nanoparticle anode for Li-ion battery with long cycle life and ultrahigh capacity" was retracted in 2023. Reasons: manipulated images; errors in the data; errors in the images; duplicated images.

# High-rate aluminium yolk-shell nanoparticle anode for Li-ion battery with long cycle life and ultrahigh capacity

**DOI:** 10.1038/ncomms8872

**Published:** 2015-08-05

**Authors:** Sa Li, Junjie Niu, Yu Cheng Zhao, Kang Pyo So, Chao Wang, Chang An Wang, Ju Li

**Affiliations:** 1 State Key Lab of New Ceramics and Fine Processing, School of Materials Science and Engineering, Tsinghua University, Beijing 100084, P. R. China; 2 Department of Nuclear Science and Engineering, Massachusetts Institute of Technology, Cambridge, Massachusetts 02139, USA; 3 Department of Materials Science and Engineering, University of Wisconsin-Milwaukee, Milwaukee, Wisconsin 53211, USA; 4 Department of Materials Science and Engineering, Massachusetts Institute of Technology, Cambridge, Massachusetts 02139, USA

## Abstract

Alloy-type anodes such as silicon and tin are gaining popularity in rechargeable Li-ion batteries, but their rate/cycling capabilities should be improved. Here by making yolk-shell nanocomposite of aluminium core (30 nm in diameter) and TiO_2_ shell (∼3 nm in thickness), with a tunable interspace, we achieve 10 C charge/discharge rate with reversible capacity exceeding 650 mAh g^−1^ after 500 cycles, with a 3 mg cm^−2^ loading. At 1 C, the capacity is approximately 1,200 mAh g^−1^ after 500 cycles. Our one-pot synthesis route is simple and industrially scalable. This result may reverse the lagging status of aluminium among high-theoretical-capacity anodes.

## Abstract (web summary)

Aluminium offers an attractive alternative anode for lithium-ion batteries, but its practical performance falls far short of the theoretical promise. Here, the authors present a yolk-shell structured nanocomposite anode of aluminium core and titanium oxide shell which displays outstanding electrochemical properties.

Aluminium should be an attractive anode material for rechargeable Li-ion batteries for many reasons, such as low cost (∼$2,000 ton^−1^), high theoretical capacity (2,235 mAh g^−1^ if Li_9_Al_4_ (refs 1, 2)), low potential plateau (∼0.19–0.45 V against Li^+^/Li^3^), high electrical conductivity and so on. However, despite the historical efforts on developing Al-Li electrodes, the practical performance fell far short of the theoretical promise and many other high-capacity anodes^3^. The best result so far came from Park *et al.*,^4^ whose hybridized 40 wt % Al/C_60_ anode showed a capacity of >900 mAh g^−1^ over 100 cycles. Most of the batteries using aluminium films of micron thickness displayed a high initial capacity, but faded rapidly in a few cycles. Fundamentally this is because of two damage mechanisms, both exacerbated by aluminium’s ∼100% volume expansion^5^/shrinkage during lithiation/delithiation: (a) the volume changes cause repeated breaking and re-formation of the solid-electrolyte interphase (SEI) film coating the active material^3^,^6^, making Coulombic efficiency (CE)≠100% in a cycle and converting cycleable or ‘live’ lithium in the electrodes and electrolyte to ‘dead lithium’ in SEI, and eventually the battery dies out of lithium exhaustion, and (b) the active material (Al-Li) could pulverize or be pushed away during cycling, thus losing electrical contact from the current collector.

The above are actually generic problems for all high-capacity anode materials^1^,^7^,^8^. Many pioneering works have shown that a predefined void space and/or a conductive buffer can counteract failure mechanisms (a) and (b)^9^,^10^,^11^. Cui *et al.,* demonstrated that creating yolk-shell nanoarchitectures^12^,^13^ could be a very effective solution, as an inert nanoshell facing the electrolyte is covered with SEI but does not change volume, while the active yolk expands/shrinks in the internal cavity without SEI. Also, because the thin carbon shell conducts both Li^+^ and electron^14^, even if the yolk pulverizes, the active contents are still confined in the closed shell and will not lose electrical contact. Ultrahigh capacity and long cycle life have been realized in the Si yolk-carbon shell electrode^7^,^12^. We believe this general paradigm should also work for aluminium active core. The key practical question is how to generate fully closed TiO_2_ nanoshell^14^ around aluminium nanoparticles with tunable vacuum interspace in between (Al@TiO_2_) in a cost-effective and industrially scalable way. From materials design point of view, the Al@TiO_2_ yolk-shell nanostructure must satisfy the following requirements: (A) The shell must be thin enough, as size-dependent transport^14^ makes thicker TiO_2_ shell a much poorer electron and Li^+^ conductor^15^. Modelling shows that sub-10 nm TiO_2_ shell has definite advantage over thicker TiO_2_ shells in transport^14^. And since TiO_2_ has a much lower capability of lithium storage than aluminium, thinner shells mean higher specific capacity of TiO_2_-nanoaluminum hybrid. Practically we are talking about TiO_2_ shell thickness *h*≤5 nm for effective transport. (B) The shell must be mechanically robust, as internal stress will still be generated within one yolk-shell due to adhesion between Al-Li core and TiO_2_ shell during lithiation/delithiation, and we do not want the thin shell to fracture in tension. Requirement (A) appears to be opposite to requirement (B), because too thin *h* clearly cannot sustain tensile load without rupturing, and too thick *h* works against transport requirement (A). But coming to the rescue, there is strong evidence that nanoscale oxides have fundamentally different mechanical behaviour from its macroscale counterpart^16^,^17^, and can be surprisingly robust mechanically^8^,^18^,^19^. So *h* of a few nanometres appears to work well enough to satisfy both (A) and (B) requirements. (C) The shell must be fully closed. This is because otherwise the liquid electrolyte can get into the void interspace by convection and generate SEI directly on aluminium surface, which triggers failure mode (a). Also, if the yolk pulverizes and the shell is not closed, the active content can spill into the electrolyte, triggering failure mode (b). (D) There must be sufficient void spacing between the yolk and shell. Since volume expansion of aluminium is ∼96%, the shell-enclosed volume (π*D*^3^/6, where *D* is the inner diameter of the TiO_2_ shell) must be at least double that of the aluminium nanoparticle (π*d*_0_^3^/6, where *d*_0_ is the diameter of the aluminium yolk before lithiation). Practically:



where we find the optimal fill factor *B* to be 2.5–4. Still larger *B* would reduce the volumetric specific capacity of Al@TiO_2_ and increase the diffusion distance, which would lead to a larger overpotential and poorer rate performance of the electrodes^20^.

In this work we report a one-pot synthesis method that is simple, cheap, scalable and uses only Earth-abundant elements (Al, Ti, O, H, C and S) and therefore can be used for mass production. The method gives specific capacities (defined based on the total weight of Al@TiO_2_ nanocomposite, or ATO powder) shown in the Abstract at an industrially sensible loading of 3 mg Al@TiO_2 _cm^−2^ on copper foil. The synthesis method is derived somewhat serendipitously. It started from the observation that some commercial aluminium powders come with a relatively thick adherent surface oxide layer of Al_2_O_3_ (alumina). Even though an ultrathin alumina membrane (by atomic-layer deposition) on high-capacity anodes could enhance performance^19^,^21^, such a thick layer of natural alumina worsens battery performance and needs to be removed. However, even if some chemical methods could be utilized to eliminate the natural alumina layer, in air, the fresh aluminium will be oxidized again very quickly. It would be great if we can design a wet-chemical environment in which the thick, adherent natural alumina layer can be converted to the beneficial, non-adherent TiO_2_ shell envisioned in (A)-(D) in just one step, to create the Al@TiO_2_ yolk-shell structure (ATO) for air-stable and long-cycle-life anode. In other words, in one stroke we would like to convert the ‘bad’ oxide (thick adherent alumina) to the ‘good’ oxide (partially detached TiO_2_ shell). By making yolk-shell nanocomposite of aluminium core and TiO_2_ shell, with a tunable interspace, we achieve 10 C charge/discharge rate with reversible capacity exceeding 650 mAh g^−1^ after 500 cycles. At 1 C, the capacity is around 1,200 mAh g^−1^ after 500 cycles.

## Results

### Preparation of Al@TiO_2_ yolk-shell nanoparticles

The chemistry for the ‘wet conversion’ has been found, which is water-based sulfuric acid ([H^+^]=1 M) saturated with titanium oxysulfate (TiOSO_4_), where the concentration of TiOSO_4_ (aq) is at the solubility limit of solid TiO(OH)_2_ that sat at the bottom of the acid bath and later filtered out:



The schematic is shown in Fig. 1a. Then, we simply place commercial aluminium powder (diameter *D*_0_∼50 nm), which have a surface layer of natural alumina, into the acid. The following ‘water-shift’ reactions (3) and (4) then take place:



where alumina is converted into aluminium sulfate (soluble) that diffuses away, and extra water. The extra water then shifts the thermodynamic balance of (2) to its right-hand side



and precipitates out solid TiO(OH)_2_ nanoshell *in situ*, by nucleation and growth at the original diameter *D*_0_. Since alumina is being consumed and the original particle recedes, the TiO(OH)_2_ solid shell at *D*_0_ starts to detach from the original particle at this point. Once alumina is completely consumed, reaction (5) takes place:



which further separates the yolk and the shell, and the interspace grows. Experimentally, we discovered reaction (5) happens slowly, on the timescale of hours. This slow etching of aluminium nanocore when there is plenty of acid in the solution proves that by the time Al_2_O_3_ is gone, the TiO(OH)_2_ shell is already fully enclosed and semi-protective, preventing the bulk acid from flowing inside by convection. But the solid TiO(OH)_2_ still allows H^+^, SO_4_^2−^, Al^3+^ ions to exchange through the shell, probably through grain boundary diffusion. So a grain boundary diffusion controlled instead of convection-controlled kinetics governs the continuous etching of aluminium yolk. The time it takes to form TiO(OH)_2_ nanoshell in acid is nearly instantaneous, so practically all of our wet-processing time is spent on reaction (5), and this time duration *t*_etch_ is our prime optimization variable, because it controls the fill factor *B* in requirement (D). For near-optimal battery performance with commercial aluminium powder (diameter *D*_0_∼50 nm), we found that *t*_etch_=4.5 h gives overall the best result (discussed below), at which point we harvest the Al@TiO(OH)_2_ powder by vacuum filtering.

We then calcine Al@TiO(OH)_2_ powder in argon to get the final Al@TiO_2_ yolk-shell (ATO) powder, during which the shell would shrink a bit. To optimize this step, TG-DSC analysis is carried out and the result is shown in Supplementary Fig. 1. The TiO(OH)_2_ shell first undergoes dehydration with a weight loss of ∼6% at a temperature of 100–300 °C. Then with continuously heating, negligible weight loss could be observed, while two exothermic peaks and one endothermic peak appear, which belong to phase transformations of amorphous TiO_2_ to anatase (395 °C), anatase to rutile (560 °C) and aluminium melting (480 °C), respectively. On the basis of the TG-DSC result, the annealing temperature we used in this study is 450 °C in argon for 1.0 h, with a heating rate of 10 °C min^−1^. This will give us anatase TiO_2_ shell. Except for the calcination, all processing steps are carried out at room temperature exposed to normal air; the entire process is industrially scalable with minimal infrastructure requirement, and the powder product is fully compatible with current slurry coating technology for battery assembly.

The interspace is adjustable through controlling the wet reaction time *t*_etch_ because a sufficient and well-defined internal void space is necessary to get an optimal performance of the ATO anode, as discussed in (A)-(D). To explore the critical experimental parameters, we synthesized ATO with different *t*_etch_. Figure 1b and Supplementary Fig. 2a reveal the X-ray diffraction patterns of the samples with different etching time. It can be seen that the original Al_2_O_3_ layer is completely eliminated after our experimental procedure and the final product consists of pure aluminium and anatase, which also indicates that the outer TiO_2_ was able to protect inner Al from being oxidized because we do not see any Al_2_O_3_ peaks (Fig. 1b). Supplementary Fig. 2b demonstrates the aluminium weight percentage for samples of different etching time determined by inductively coupled plasma analysis, and Supplementary Fig. 2c shows the corresponding specific capacity at 1 C. Overall, for samples with such high aluminium percentage (85 wt %), a remarkable battery performance is observed. For *t*_etch_=3.0 h, the capacity is as high as 1,400 mAh g^−1^ at 1 C at 300 cycles. Severe capacity fading is observed after 300 cycles, which is believed to be due to the insufficient void space (*B*∼2, Supplementary Fig. 2c, red and Supplementary Fig. 11). After hundreds of cycles, the Al-Li yolk will finally rupture the TiO_2_ shell. Then, repeated unstable SEI formations ensue. In contrast, for the sample with longer *t*_etch_=4.5 h, the initial reversible capacity is a little bit lower than the former one due to smaller yolk-to-shell weight ratio, but the performance is ultra-stable in the whole 500 cycles, illustrating the compromise between transport and mechanical considerations (A), (B), (D) in materials design. Comparing the four results, the optimal *t*_etch_ is determined to be 4.5 h, corresponding to *d*=30–35 nm and *D*_0_=47 nm (measured from transmission electron microscopy (TEM)), and *B*=2.4–3.8.

Figure 2a shows SEM image of the as-obtained Al@TiO_2_ yolk-shell particles with *t*_etch_=4.5 h, which clearly reveals a solid core encapsulated by a nearly spherical shell (arrows). However, it is worth mentioning that the starting aluminium nanoparticles often stick together even after sonication, and so double-yolk single-shell or even multiple-yolk single-shell structures are also obtained after reacting with acid (Supplementary Fig. 3), which does not seem to degrade the performance much. Energy-dispersive X-ray spectrum (Supplementary Fig. 4) of the nanostructure in Supplementary Fig. 3a demonstrates the presence of Al and TiO_2_. TEM results indicate a complete coverage of TiO_2_ (Fig. 2b), which is crucial for blocking the electrolyte convection and limiting SEI formation to the outer shell surface. Inside, aluminium nanoparticles, about *d*=30–35 nm in diameter, are encapsulated by the TiO_2_ shell, with well-defined void space in between that can accommodate the volume expansion. The TiO_2_ framework, although only a few nanometres thick, was able to firmly support the core (design requirement (B)) and semi-effectively protect the chemically active aluminium (as revealed in Supplementary Fig. 5). Here we would like to reiterate the three purposes of the TiO_2_ shell: first, during the acidic material preparation process, it protects the as-formed fresh aluminium particles in the core; moreover, the TiO_2_ shells not only work as a conducting framework^14^,^15^, but also as an electrolyte blocking layer, so SEI forms outside the shell. The element mapping in Fig. 2d–f further confirms the yolk-shell characteristic with aluminium as the core, TiO_2_ as the shell and the void in between.

### Half-cell battery performance of Al@TiO_2_ yolk-shell nanoparticles

The Al@TiO_2_ yolk-shell nanocomposite exhibits remarkable battery performance. As shown in Fig. 3a, at a rate of 1 C, the first discharge and charge capacities are 1,237 and 1,360 mAh g^−1^, respectively, which indicate a first-cycle CE of 90.9%. (The 9.1% unbalanced charge-discharge electrons, or ‘AWOL electrons’, in the first cycle mostly likely reflect the asymmetric formation of SEIs covering the two electrodes). Then, the specific capacity stabilizes at 1,170 mAh g^−1^ in later cycles. Importantly, the Al@TiO_2_ yolk-shell powder has long cycle life and the capacity decay is only<0.01% per cycle. The average CE is 99.2% in the first 500 cycles. The voltage profiles for the different cycles are shown in Fig. 3b. The shape of the profile does not change from the 250th to the 500th cycle, indicating ultra-stable performance. At rate 10 C, the Al@TiO_2_ yolk-shell electrode can still achieve a capacity of 661 mAh g^−1^ after 500 cycles, twice the capacity of graphite as shown in Fig. 3c,d. We believe the excellent rate performance of ATO is due to aluminium’s good electrical conductivity, which is an advantage over Silicon as the active material. This high performance persists to 750 cycles (Supplementary Fig. 10), even though faster capacity decay (∼0.03% per cycle) appeared after the 500th cycle or so. Given that the SEI layer may have time-dependent growth, a slow cycling rate of 0.1 C was checked, as shown in Supplementary Fig. 8, and an even higher reversible capacity of 1,599 mAh g^−1^ was achieved for 100 cycles.

Figure 4 shows the structure of Al@TiO_2_ yolk-shell after 500 charge-discharge cycles. We see that the yolk-shell stays intact even after 500 cycles, which explains the good cyclability. The shell’s outer surface becomes thicker and rougher after the battery test, indicating the formation of the SEI layer on the TiO_2_ shell. (The electrochemical stability window of the ethylene carbonate—diethyl carbonate electrolyte used in this study is 1.3–4.5 V versus Li^+^/Li, so SEI will form when the cycling voltage drops below 1.3 V.) The elemental mapping in Fig. 4d–f also reveal a perfect yolk-shell structure after 500 cycles, and therefore we can conclude that the void between the yolk and shell has successfully accommodated the volume expansion/shrinkage during the many cycles, satisfying design principles (A) and (B). We believe design principle (C) is also satisfied throughout, that is, the shell stays fully enclosed, because otherwise the SEI debris from the reactions with the electrolyte would have filled out the inside of the cavity like for other Al-based anodes^22^. To be able to cycle 500 times with a pristine interior surface means the shell integrity is excellent. Supplementary Fig. 9 shows the X-ray diffraction pattern of Al@TiO_2_ anode at 0th, 15th and 510th cycle. Compared with the initial crystalline Al FCC structure, we see the nanoaluminum inside has turned amorphous. In (ref. 23), elemental metals tens of nanometres in domain size has turned amorphous under rapid temperature quenching. We believe electrochemical shock^17^ could have similar effect of solid-state amorphization^24^.

Cyclic voltammetry was performed on ATO (Supplementary Fig. 12). During the cathodic scan, the cell displayed a well-defined peak potential at 0.23 V and a prominent peak potential at 0.50 V was observed in the anodic sweep, which correspond to the discharging and charging plateau in Fig. 3b, respectively, representing the alloying/dealloying of aluminium. Meanwhile, one pair of broad cathodic/anodic peaks (located at 1.68 and 1.89 V) corresponding to Li-insertion/extraction in TiO_2_ could also be detected, suggesting a pseudocapacitor-like characteristic of TiO_2_ shells during lithiation and delithiation. For the sake of comparison, completely hollow TiO_2_ (without Al) was synthesized using an etching time of 24.0 h (Supplementary Fig. 6) and its cycling performance at 1 C was also characterized (Supplementary Fig. 7). The reversible capacity of hollow TiO_2_ particles reaches 112 mAh g^−1^ for the first cycle and stabilizes at 111 mAh g^−1^ for later cycles. Moreover, it is interesting to find that the hollow TiO_2_ nanoshells exhibit a quasi-linear voltage–capacity response (instead of a voltage plateau) during galvanostatic charging-discharging, consistent with the broad cyclic voltammetry peaks at 1.68 and 1.89 V. We believe the reason for such pseudocapacitive behaviour is that when the TiO_2_ shell (∼3 nm) is extremely thin, a large fraction of lithium storage sites are on the surface or in near-surface regions^25^. After deducting the TiO_2_ contribution, the specific capacity with respect to nanoaluminum is calculated to be 1,246 mAh g^−1^ at 1 C.

### Full-cell performance against Li-matched LiFePO4 cathode and Coulombic efficiency

All the tests above were performed with half-cells, where the counter-electrode used was lithium metal with super-abundant moles of lithium (∼1,000%) relative to the ATO capacity. Half-cell tests are known to be unreliable checks of failure mechanism (a). Passing the more rigorous full-cell tests, where one uses lithium-molar-matched counter-electrode, would certify ATO as being close to practical use. Therefore, we have fabricated full cells with ATO anode, and LiFePO_4_ (LFP) cathode with only 35% more lithium relative to the ATO capacity in half-cells. The fact that metallic lithium foil is no longer used, which served both as an abundant Li-ion source and as a reference electrode with little potential change on lithiation/delithiation, critically tests the applicability of ATO in a real-world context. Even after including all lithium ions contained in the electrolyte salt, the total lithium contained in our full cells does not exceed ∼150% of the ATO capacity. Supplementary Fig. 13 shows our full cell exhibited a first discharge capacity of 1,123 mAh (g of ATO)^−1^ at a rate of 1 C from 2.5 to 4.0 V, with a first-cycle CE=79.4%. This means in the first cycle, >20% within the ∼50% excess lithium was used to form initial SEI that cover the large surface area of Al@TiO_2_ yolk-shells. This is normal and common treatment in all commercial batteries. The key question is from the second cycle on, whether the remaining <∼30% excess lithium is sufficient to sustain large number of cycles. Supplementary Fig. 13 shows that it indeed does: the specific capacity stabilizes at ∼968 mAh (g of ATO)^−1^ up to 200 cycles in the full cell. This proves that the TiO_2_ shells are indeed robust enough that a great majority of the Al@TiO_2_ yolk-shell survives, and that the SEI is stable outside of TiO_2_.

Curiously, our full-cell tests showed an average CE of only 99.48% from the 2nd to 200th cycles. Even though our ATO’s CEs in half-cell and full-cell tests are actually very good compared with most of the high-capacity electrodes in the literature, it seems to violate a commonly held belief of the battery industry that the Coulombic efficiency needs to exceed 99.9% to be able to cycle 200 times, since (0.999)^200^=0.82, and 80% capacity retention is a typical definition of battery life. Our full-cell tests prove that the Coulombic efficiency does not have to be >99.9% in order for lithium-matched full cells to cycle 200 times. We believe this is because the unbalanced charge-discharge electrons (AWOL electrons) do not all tie down Lithium irreversibly. Here we believe the 0.52% absence without leave (AWOL) electrons are not all generating irreversible SEI, but instead forming reversible redox shuttle inside the electrolyte, as illustrated in Supplementary Fig. 14 (ref. 26). This is probably water-related, since it is hard to make our ATO completely dry, and a possible chemical mechanism involving hydrogen radical transport is proposed in Supplementary Note. To double check, we directly estimated the total mass of SEI on ATO by measuring the mass of ATO based anode after 50, 100, 150 and 200 cycles. There is only ∼40% mass increase relative to the initial ATO weight (without binder and carbon black) after 200 full-cell cycling, shown in Supplementary Fig. 15, which is much better than previous Al-based anodes, where the SEI debris is seen to completely bury the Al^22^. If the AWOL electrons indeed were all used to form SEI or other irreversible products that tie down Li irreversibly and forever, then there is no way that 85.3% capacity retention was maintained in this lithium-matched full cell after 200 cycles, since 0.52% × 200>100%, and utter lithium exhaustion is predicted.

We contrast ATO with existing anode technologies. Compared with metallic lithium, ATO does not form dendrites at high rate and is less of a safety concern because of air stability. Compared with Si yolk-carbon shell^7^, ATO has ∼20% lower capacity below 1 C rate, but provides higher capacity with long cycle life above 1 C. Compared with high-rate Li_4_Ti_5_O_12_ anode which has extremely long cycle life, ATO has 8 × gravimetric capacity at 1 C, and much better (lower) voltage. Compared with conventional graphite anode (theoretical capacity 372 mAh g^−1^) used in current batteries, ATO has similar voltage characteristics, but has 4 × gravimetric capacity at 1 C charge/discharge rate. The fact that ATO achieves 10 C charge/discharge rate with reversible capacity exceeding 650 mAh g^−1^ even after 500 cycles makes it a high-rate and ultrahigh-capacity anode, at an industrially satisfactory loading of 3 mg cm^−2^. Simple and scalable nanostructuring has thus realized the intrinsic potential of this abundant element for battery anode.

## Discussion

In summary, we developed a scalable, low-cost synthesis of Al/TiO_2_ yolk-shell nano-architecture (ATO) using a wet-chemical method. The nano-scaled framework is composed of a solid Al core with a adjustable interspace, and a titanium oxide layer, which can suppress Al oxidation but not impairing electrochemical activity. The assembled half-cell using Nano-ATO as anode exhibited a long cycle life and an admirable rate capability. A largely improved capacity of ∼1,200 mAh g^−1^ along with an average CE of ∼99.2% over 500 cycles at 1 C was achieved. Moreover, owing to the high Li^+^/electron conductivity of Al and TiO_2_, a capacity of 661 mAh g^−1^ still remained after 500 cycles at a fast rate of 10 C. Full-cell tests against LFP cathode with only 35% excess Lithium were successful for 200 cycles, verifying that ATO is close to real applications, as anode for high energy- and power-density Li-ion batteries.

## Methods

### Synthesis of Al@TiO_2_ nanoparticles

Al@TiO_2_ was synthesized using an ‘*in situ* water-shift’ method (See Full Method in Supplementary Methods). Specifically, 0.05 g TiOSO_4_ (reagent grade, Sigma-Aldrich) and 3.0 g H_2_SO_4_ (ACS grade, 1.0 N, VWR) were dissolved in 100 ml deionized water. Then, 0.135 g Al powder (∼50 nm in diameter, 99.9%, US Research Nanomaterials, Inc.) was added to the saturated TiOSO_4_ solution. After the 30 min vigorous agitation using an ultrasound cleaner (Symphony, VMR), the solution was stirred for 3.0–10.0 h until the colour changed from grey to light. Then the resultant solution was filtrated in a vacuum system and washed three times by ethanol. After drying at 70 °C for 7.0 h in a vacuum oven (Symphony, VMR), the sample was annealed at 450 °C for 1.0 h in an Ar filled quartz tube furnace (Lindberg Blue M, Thermo Scientific). Finally, the sample was collected for the characterization and battery test.

### Characterization

X-ray diffraction measurements were carried out via a Bruker D8-Advance diffractometer using Ni filtered Cu Kα radiation. SEM images were collected on a FEI Sirion scanning electron microscope and TEM images were taken on a JEOL JEM-2010 transmission electron microscope operated at 200 kV. TG-DSC analysis was performed using Netzsch STA 449 with air flow at a heating rate of 10 °C min^−1^ from room temperature to 600 °C. Inductively coupled plasma mass spectrometry was carried out using a Thermo Scientific ICAP 6300 Duo View Spectrometer. (See details in Supplementary Methods).

### Electrochemical test

The battery performance of Al@TiO_2_ as anode was measured using a coin cell (CR2032, Panasonic). The ATO electrode was prepared by mixing the Al@TiO_2_ (70 wt %), 15 wt % conductive carbon black (Super C65, Timcal) and 15 wt % poly(vinylidene fluoride) binder (Sigma-Aldrich) in N-methyl-2-pyrrolidinone solvent (Sigma-Aldrich). The obtained slurry was coated on copper foil with a loading of 3 mg cm^−2^ of Al@TiO_2_ and dried at 65 °C for 24.0 h. The half-coin cell using a Li foil as a counter and reference electrode was assembled in a glove box (Labmaster sp, MBraun) filled with argon. To suppress lithium dendrite formation and also improve the cycle performance of the lithium foil in half-cell, a Li_3_N passivation layer was coated on the lithium foil electrode before battery assembly. The pretreatment procedure exposes one face of a fresh Li foil (thickness ∼600 μm) to flowing N_2_ gas at a constant velocity for 2 h at room temperature to form Li_3_N. When preparing the half-cell, the pretreated side of lithium foil would be in contact with the electrolyte. A hydraulic crimping machine (MSK-110, MTI) was used to close the cell. The electrolyte was 1.0 M LiPF_6_ dissolved in 1:1 (volume) ethylene carbonate and diethyl carbonate, and a microporous polyethylene film (Celgard 2400) as the separator. The assembled cell was cycled between 0.06 to 2.0 V at various rates ranging from 0.1 to 10 C by a LAND 2001 CT battery tester. All of the specific capacities were calculated on the basis of total mass of Al@TiO_2_ except the data in Supplementary Table 1 and Supplementary Fig. 10b were based on pure aluminium. The C rate was calculated on the basis of theoretical capacity 1,410 mAh g^−1^ of Li_3_Al_2_. The cyclic voltammetry curves were obtained at room temperature using the coin cells above between 0.06 and 2 V at a scan rate of 0.1 mV s^−1^. Full cells consisting of ATO as the anode, LFP as the cathode, and a 1 M LiPF_6_ EC:DEC 1:1 solution as the electrolyte were fabricated and tested. The ATO anode was prepared using the same method described above and the electrode film was punched into discs with diameter of 10 mm before battery assembling in a glove box filled with argon gas. The LFP electrodes were fabricated by spreading the mixture of LFP (Pulead Technology Industry Co., Ltd.), carbon black (Super C65, Timcal) and poly(vinylidene fluoride) binder (Sigma-Aldrich) with a weight ratio of 80:10:10 on Al current collectors. The electrode was pressed under 6–10 MPa and punched into 11 mm diameter circular disks. The active material loading was 1.3 mg cm^−2^ for the ATO anode and 10.5 mg cm^−2^ for the LFP cathode. The mass of ATO, LFP and even the lithium salt in the electrolyte was carefully calculated/weighed, and the total lithium contained in our full cells does not exceed ∼150% of the ATO capacity in half-cell. The matched ATO/LFP full cells were evaluated by galvanostatic cycling in a 2,032 coin-type cell at 2.5–4.0 V, 1-C rate (1,410 mA g^−1^ of ATO). The mass of SEI layers is estimated by measuring the mass of ATO active materials based anode before and after 50, 100, 150 and 200 cycles. The normalized mass of SEI is defined as the ratio of the mass gain on ATO after cycling (presumably due to SEI layers covering ATO) to the initial ATO mass loaded in the cell without SEI. Two LFP/ATO full cells were used for the average normalized mass of SEI for each cycling condition. (See details in Supplementary Methods).

## Additional information

**How to cite this article:** Li, S. *et al.* High-rate aluminium yolk-shell nanoparticle anode for Li-ion battery with long cycle life and ultrahigh capacity. *Nat. Commun.* 6:7872 doi: 10.1038/ncomms8872 (2015).

## Supplementary Material

Supplementary Information Supplementary Figures 1-15, Supplementary Table 1, Supplementary Notes, Supplementary Methods and Supplementary References

## Figures and Tables

**Figure 1:** Synthesis and characterization of Al@TiO_2_. (**a**) Schematic of the ‘*in situ* water-shift’ synthesis of Al@TiO_2_. The colours represent chemical contents in the solution: the equilibrated mixture of H_2_SO_4_ and TiOSO_4_ is light yellow, H_2_O is blue, and H_2_SO_4_ is green. (**b**) X-ray diffraction data of commercial nano aluminium powder and the as-obtained Al@TiO_2_ with 4.5 h etching. The original Al_2_O_3_ layer is completely eliminated after our experimental procedure and the final product consists of pure metallic aluminum and anatase.

**Figure 2:** Morphology analysis of the as-obtained Al@TiO_2_ with etching time of 4.5 h. (**a**) SEM image of Al@TiO_2_ with a broken shell. Bright-field transmission electron microscopy images of Al@TiO_2_ at (**b**) low and (**c**) high magnifications, indicating the inner aluminum yolk encapsulated by the TiO_2_ shell. Scale bars, **a** and **b**, 20 nm; **c**, 10 nm. The chemical composition was confirmed by the element mappings of (**d**) Ti, (**e**) O, and (**f**) Al, corresponding to the structure shown in (**c**).

**Figure 3:** Half-cell battery performance of Al@TiO_2_ (4.5 h etching). (**a**) Cycling life and the corresponding Coulombic efficiency during 500 cycles. The charge/discharge rate was set at 1 C. (**b**) Charge/discharge voltage profiles with the 1st, 250th and 500th cycling. (**c**) Cyclability test at different charge/discharge rates. (**d**) Delithiation capacity evolution by varying charge/discharge rates ranging from 0.1, 0.5, 1, 2, 5, 10 C and back to 0.1 C.

**Figure 4:** Morphology evolution of Al@TiO_2_ after the coin cell was tested 500 cycles. (**a**) a SEM and (**b**,**c**) bright-field transmission electron microscopy images of Al@TiO_2_, showing the Al/TiO_2_ yolk-shell structure was still well maintained after 500 cycles. Scale bars, **a** 50 nm; **b** and **c**, 20 nm. The chemical element mappings of (**d**) Ti, (**e**) O, and (**f**) Al, corresponding to the structure shown in (**c**), was confirmed by Energy-dispersive X-ray spectroscopy (EDS).
